RETRACTED

# Exploration on Molecular Mechanism of Reversal Effect of Compound Danshen Tablets on Hepatic Fibrosis Based on Network Pharmacology

**DOI:** 10.1155/2022/7241719

**Published:** 2022-05-10

**Authors:** Minling Cao, Jingyue Fan, Xiaoli Yang, Meifeng Shi, Shanshan Lin, Xiaoling Chi

**Affiliations:** Department of Hepatology, The Second Affiliated Hospital of Guangzhou University of Chinese Medicine, Guangdong, Guangzhou 510007, China

## Abstract

**Objective:**

To research the molecular mechanism of compound Danshen tablets in the treatment of hepatic fibrosis through network pharmacology.

**Methods:**

Traditional Chinese medicine systems pharmacology (TCMSP) and online Mendelian inheritance in man (OMIM) databases were searched for compound Danshen tablets' active ingredients o and hepatic fibrosis-related genes. The network enrichment of the targets of “herb-compound-target” was visualized and analyzed using Cytoscape software. Then, the screened target genes were used to construct a protein-protein interaction network. The DAVID enrichment database (the database for annotation, visualization, and integrated discovery) was adopted for GO (Gene Ontology) enrichment and KEGG (Kyoto Encyclopedia of Genes and Genomes) pathway enrichment of vital nodes.

**Results:**

The results yielded 234 targets of compound Danshen tablets; ten important targets (TNF, IL-10, TGF-*β*1, EGF, CXCL16, CCL21, SERPINB5, SERPINA1, SOD2, and PPIG) for reversing hepatic fibrosis; and four core targets (TNF, IL-10, TGF-1, and EGF). In addition, KEGG enrichment analysis showed that compound Danshen tablets mainly involved FoxO and MAPK signaling pathways, as the key signaling pathways in the treatment of hepatic fibrosis.

**Conclusion:**

TNF, IL-10, TGF-1, and EGF and FOXO and MAPK signaling pathways play a key role in the pathogenesis of hepatic fibrosis. Based on the results of this study, the mechanism of action of compound Danshen tablets in the treatment of hepatic fibrosis may be associated with the regulation of FoxO and MAPK signaling pathways and inhibition of TNF, IL-10, TGF-1, and EGF.

## 1. Introduction

Hepatic fibrosis is associated with high morbidity and mortality. It is a complex compensatory process for tissue repair in which large amounts of extracellular matrix produced by activated hepatic stellate cells (HSCs) are deposited excessively in the liver [1]. Hepatic fibrosis can be stimulated by hepatocyte injury, inflammation, hepatotoxicity, immune complex deposition in immune response, hepatic congestion, hypoxia, cholestasis, and siderosis . While hepatic fibrosis or early cirrhosis is considered reversible [3, 4], to date, there are no clear chemical or biological antifibrotic drugs in clinical practice. Consequently, there have been research and developments efforts for effective hepatic treatment with an aim of preventing progression to cirrhosis and hepatocellular carcinoma [5].

RETRACTED

Traditional Chinese medicines have been shown to have effective therapeutic effects with minimal side effects and have been used for the treatment of a wide range of diseases including hepatopathy [6]. They have been shown to protect hepatocytes, inhibit hepatic inflammation, and reduce fibrosis. In addition, in the treatment of hepatic fibrosis, traditional Chinese medicine offers unique benefits owing to its syndrome and disease differentiation and comprehensive pharmacological effects and multichannel, multilevel, and multitarget [7, 8]. However, in some cases, traditional Chinese medicine may not treat the source of the disease (e.g., viruses that cause hepatitis) and therefore cannot replace conventional medicine [8]. In recent studies, the integrative health concept has been shown to have benefits in various situations; combinations of traditional Chinese medicines and antiviral drugs were shown to have enhanced therapeutic effects on hepatic fibrosis compared to antiviral drugs alone. Chinese traditional medicines that were used in such combinations included Anluohuaxian capsules, Fuzheng Huayu capsules/compound, and Biejia Ruangan prescription [9–13].

Traditional Chinese medicines may also be an effective prevention approach for hepatic fibrosis [14]. Additionally, with multitarget features, traditional Chinese medicines can play a role in multidirectional repair. Many Chinese patent antihepatic fibrotics have been registered and marketed for clinical application. Radix notoginseng and radix salviae miltiorrhiza are the key components of the marketed antihepatic fibrosis traditional Chinese medicines (e.g., Fuzheng Huayu capsules and Anluohuaxian capsules), and borneol is used as a messenger drug to enhance efficacy. Compound Danshen tablets which contain radix notoginseng, radix salviae miltiorrhiza, and a small amount of borneol are Chinese patent medicines commonly used in clinical practice for the treatment of coronary heart disease [15]. Some studies have shown that compound Danshen tablets combined with Xiaoyao pills can treat hepatic fibrosis effectively [16]. Besides, the compound Danshen dripping pill effectively reduced hepatic fibrosis injury in rats [17], and the reversal effect of compound Danshen injection on hepatic fibrosis has been applied in clinical practice [18]. However, while the core molecular mechanism of the antihepatic fibrosis of compound Danshen tablets is significant as it contributes to its therapeutic value, it is still unclear. Therefore, this study is aimed at investigating the molecular mechanism of compound Danshen tablets in the treatment of hepatic fibrosis through network pharmacology.

RETRACTED

## 2. Methods

### 2.1. Screening of the Compound Danshen Tablets' Active Ingredients

Compound Danshen tablets contain three traditional Chinese medicines. The Traditional Chinese Medicine Systems Pharmacology (TCMSP) database (Target information was mainly from Drug Bank) was searched for active ingredients of the three traditional Chinese medicines using the “compound Danshen tablets” as the keyword. Oral bioavailability (OB) and drug-likeness (DL) of compound Danshen tablets were used as the screening parameters of the collected active ingredients. Then, the collected active ingredients were screened according to the screening conditions and integrated model of drug absorption, distribution, metabolism, and excretion (ADME). Subsequently, based on the active ingredients screening feedback suggestions in the document “parameter information” of the Chinese TCMSP document database, the following compound screening threshold conditions were determined: bioavailability ≥ 30% and congener medicine property ≥ 0.18. The compounds' structures were searched in PubChem (https://pubchem.ncbi.nlm.nih.gov/), and then the target proteins corresponding to the compounds screened from the Pharmmapper and PubMed databases were standardized in UniProt. Then, Cytoscape 3.7.2 software was used to construct the “active compound of compound Danshen tablets-target” network.

### 2.2. Hepatic Fibrosis Disease Target Identification

Known hepatic fibrosis genes were searched through the online Mendelian inheritance in man (OMIM) database (https://omim.org/), using “hepatic fibrosis” as the keyword. The targets of Homo sapiens were selected, and “uncompressed” was chosen to download the EXL form. After reduplicated data were removed, the EXL form was added to “OMIM hepatic fibrosis database.” Then, the gene ID in “OMIM hepatic fibrosis database” was converted to pronKB by querying the UniProt database and using the plotting function. After downloading the EXL, protein name and gene name columns were sorted, and the key information was screened to obtain “hepatic fibrosis-target.” Then, the gene names in the “active compound of compound Danshen tablets-target” and “hepatic fibrosis-target” were converted into gene symbols one at a time through querying the UniProt database. After that, the target information was input in the UniProt KB column, and human was chosen from popular organisms. Then, the gene name whose weight was ranked first was used to construct the UniProt-gene name database. Subsequently, according to the type file formed, the processed data were imported into Cytoscape 3.7.2 to construct the “compound Danshen tablets-compound-target-hepatic fibrosis” network.

RETRACTED

### 2.3. Screening of Target Interaction Network of the Compound Danshen Tablets-Hepatic Fibrosis and Key Target

The gene names in the “active compound of compound Danshen tablets-target” and “hepatic fibrosis-target” were converted to gene symbols using the UniProt database. Subsequently, gene symbol information from the two databases was combined to screen for overlapping targets of the compound Danshen tablets and hepatic fibrosis. The STRING database was used to analyze all gene symbols and obtain target interaction information. In order to obtain the highest confidence level of interconnection, the node data screening was performed with “High Confidence (0.700),” and the processed gene symbol data were imported into the Cytoscape 3.7.2 software for network visualization display. After that, topology analysis was conducted according to the network diagram composited by gene symbols, and the top 10 genes were selected as key targets in the compound Danshen tablets-hepatic fibrosis network according to the ranking of the weighting exponent of the node degree. Then, the STRING database was used to analyze the target interaction information between the top 10 genes to obtain the core targets.

### 2.4. Bioinformatics Annotation

DAVID database (https://david.ncifcrf.gov) was adopted to perform Gene Ontology (Go) analysis and Kyoto Encyclopedia of Genes and Genomes (KEGG) analysis for common signaling targets of compound Danshen tablets-hepatic fibrosis. “Homo sapiens” was chosen in the gene-enriched species column. After screening, the gene enrichment results of *p* < 0.05 or FDR < 0.01 were used as output for data analysis and plotting.

## 3. Results

### 3.1. Establishment of “Compound Danshen Tablets-Target Active Ingredients” Network

TCMSP and UniProt databases were searched for active ingredients of compound Danshen tablets-target, and Cytoscape 3.7.2 was adopted to conduct network visualization processing for the data. The search yielded 57 active ingredients and 925 targets for radix salviae miltiorrhiza and 7 active ingredients and 246 targets for radix notoginseng. Borneol, as the messenger drug and active ingredient after metabolism, did not form a target in the TCMSP database query. After combination and deduplication, 234 targets of compound Danshen tablets were obtained (Figure 1). Additionally, in order to determine disease targets, hepatic fibrosis-related diseases in the OMIM database were collected, and the targets of the samples of Homo sapiens were screened; finally, a total of 162 important targets for hepatic fibrosis were obtained.

RETRACTED

### 3.2. Analysis of the Basic Targets of Compound Danshen Tablets for Antihepatic Fibrosis Effects

Target interaction information was analyzed through the STRING database. First, interaction targets were obtained by hiding independent individuals and setting high confidence levels. Then, the physical subnet network edge was replaced to obtain high-confidence interaction targets. Finally, based on the thickness and intensity of the interaction lines in a protein-protein interaction network diagram, the top 10 key targets (TNF, IL-10, TGF-*β*1, EGF, CXCL16, CCL21, SERPINB5, SERPINA1, SOD2, and PPIG) were obtained. Among the targets, the core targets were TNF, IL-10, TGF-*β*1, and EGF and the main active ingredients of compound Danshen tablets exerting antihepatic fibrosis effect included quercetin (TNF, IL-10, TGF-*β*1, and EGF), *β*-sitosterol (TGFB1), ginsenoside Rh2 (TNF) in radix notoginseng, and luteolin (TNF, IL-10, and EGF) and cryptotanshinone (TNF) in radix salviae miltiorrhiza (Figures 2(a)–2(c)).

### 3.3. GO Analysis and KEGG Pathway Enrichment

GO analysis of the common compound Danshen tablets-hepatic fibrosis targets was conducted, including biological process (BP), cell component (CC), and molecular function (MF). The data from the STRING database were searched for items of *P* ≤ 0.0163, and the top 21 pathways were selected according to the *P* values from the smallest to largest after enrichment; then, a histogram was drawn. The common compound Danshen tablets-hepatic fibrosis database targets were taken through KEGG pathway enrichment analysis and then imported into the STRING database. After that, the items of *P* ≤ 0.01 were selected; then, the top 17 pathways were screened according to the *P* values from the smallest to largest, and a histogram was drawn for literature analysis. The results of GO analysis showed that compound Danshen tablets exerted their effects through the chemokine signaling pathway, by regulation of chronic inflammatory reaction and endothelial cell apoptosis process, and cytokine-cytokine receptor interaction. In addition, KEGG enrichment analysis showed that compound Danshen tablets mainly involved FoxO and MAPK signaling pathways, as the key signaling pathways in the treatment of hepatic fibrosis (Figures 3(a) and 3(b)). The above results suggested that compound Danshen tablets treat hepatic fibrosis by regulating different biological processes.

## 4. Discussion

Network pharmacology and system biology can explain the effects of drugs on biological network disruption from the perspective of macroscopic or holistic regulation [19]. Similarly, they provide new ideas and technologies for the study of the traditional Chinese medicine compounds' mechanism of action [20]. Network pharmacology and system biology have been applied in the pharmacodynamic evaluation and drug mechanism of action research [21]. Traditional Chinese medicines have multiple advantages based on their multiple target ability as one of their therapeutic mechanisms and have consequently become an important antihepatic fibrosis approach in recent years. In addition, the multitargeted pathogenesis of hepatic fibrosis provides an added advantage to traditional Chinese medicines in the treatment of hepatic fibrosis. Besides containing radix notoginseng and radix salviae miltiorrhiza (two core components in the marketed anti-hepatic fibrosis medicines), a small amount of borneol was also added in compound Danshen tablets as a messenger drug to enhance antifibrosis effects. As shown by the enrichment analysis results, TNF, IL-10, TGF-*β*1, EGF, CXCL16, CCL21, SERPINB5, SERPINA1, SOD2, and PPIG were the important targets, and TNF, IL-10, TGF-*β*1, and EGF were the major core targets for compound Danshen tablets in reversing hepatic fibrosis. Besides, the corresponding drug-active ingredients of compound Danshen tablets included quercetin (TNF, IL-10, TGF-ß1, and EGF), *β*-sitosterol (TGFB1), and ginsenoside Rh2 (TNF) in radix notoginseng and luteolin (TNF, IL-10, and EGF) and cryptotanshinone (TNF) in radix salviae miltiorrhiza. The above core targets promoted hepatic fibrosis by cytokine-cytokine receptor interaction, regulation of antigenic stimulation on chronic inflammatory reaction, biosynthesis of the receptors, endothelial cell apoptosis process, chemokine signaling pathway, and regulation of hyaluronan biosynthesis [22, 23]. Further, several reviews have emphasized the key role of hepatic stellate cell and myofibroblasts' activation in the pathogenesis of hepatic fibrosis; the activation is mediated by cytokines and chemokines. TGF-b1 stimulates its own production by myofibroblasts, consequently establishing an autocrine cycle of myofibroblast differentiation and activation [24]. TNF*α* can trigger multiple signaling pathways involved in inflammation; further, TNF*α* production perpetuates the inflammation phase which results in the activation of resident HSCs into fibrogenic myofibroblasts [25]. IL-10 exerts fibrogenic effects through macrophages; exogenous IL-10 inhibits mmp-9 (92-kda gelatinase) synthesis and blocks LPS-stimulated mmp-1 expression by human macrophages while it stimulates their TIMP-1 production [26]. EGF, the epidermal growth factor, can stimulate and promote the formation and growth of various epidermal and epithelial tissues in vivo and stimulate the growth of some fibroblasts in cell culture [23]. The FoxO subfamilies belong to the forkhead box transcription factor family. FoxO subfamilies are involved in the regulation of cell anabolism, inter-conversion, survival, migration, and proliferation. Currently, there are four homologous genes of FoxO found in the genes of Homo sapiens: FoxO1, FoxO2, FoxO3a, and FoxO4. Among the homologous genes [27], FoxO1 is a core transcription factor in hepatic fibrogenesis, which affects the activation, proliferation, and migration of HSCs and participates in the process of hepatic fibrosis progression. Mitogen-activated protein kinase (MAPK) is a signal transduction pathway that has received great attention in recent years. MAPK, as a relatively mature and classical signaling pathway, mainly plays its role through a series of intracellular biological stimuli. Specifically, an intracellular biological stimulus occurs when an extracellular receptor stimulates a signal source and transmits molecules into the entire nucleus [28]. The MAPK signaling pathway is the “messenger” through which the extranuclear signals enter the nuclear interior via the transduction pathway. Notably, the dynamic changes of proteins in the MAPK signaling pathway have attracted increasing attention. At the present, it is believed that the MAPK signaling pathway regulates the development of hepatic fibrosis and cirrhosis in many aspects, such as the regulation of chronic inflammatory reaction, cell cycle apoptosis process, and cytokine interaction.

RETRACTED

Taken together, these results suggest that, possibly, inhibition of the four core targets (TNF, IL-10, TGF-1, and EGF) and FOXO and MAPK signaling pathways by the compound of Danshen tablets could result in reversal effects on hepatic fibrosis.

## 5. Conclusion

TNF, IL-10, TGF-1, and EGF and FOXO and MAPK signaling pathways play a key role in the pathogenesis of hepatic fibrosis. Therefore, the mechanism of action of compound Danshen tablets in the treatment of hepatic fibrosis may be associated with the regulation of FoxO and MAPK signaling pathways and inhibition of TNF, IL-10, TGF-1, and EGF. Further, the development of TNF, IL-10, TGF-ß1, and EGF receptor antagonists could be an effective therapeutic approach to hepatic fibrosis.

## Figures and Tables

**Figure 1:** Network diagram of the compound Danshen tablets targets.

**Figure 2:** Analysis of the basic targets of compound Danshen tablets for anti-hepatic fibrosis effects. Interaction targets obtained by hiding independent individuals, setting high confidence level (a) and replacing physical subnet network edge (b) in STRING database; (c) top 10 key targets obtained based on the thickness and intensity of the interaction lines in protein-protein interaction network diagram.

RETRACTED

**Figure 3:** GO and KEGG pathway enrichment analysis for the common targets of compound Danshen tablets for hepatic fibrosis treatment. Go (a) and KEGG pathway enrichment analysis (b) for common targets of compound Danshen tablets for hepatic fibrosis treatment.

## Data Availability

The data used to support the findings of this study are available from the corresponding author upon request.
